The article "Mass–Energy Equivalence Extension onto a Superfluid Quantum Vacuum" was retracted in 2021. Reasons: concerns about the data; concerns about the results or conclusions; concerns about the citations.

# Mass–Energy Equivalence Extension onto a Superfluid Quantum Vacuum

**DOI:** 10.1038/s41598-019-48018-2

**Published:** 2019-08-13

**Authors:** Amrit Srečko Šorli

**Affiliations:** Bijective Physics Institute, Idrija, Slovenia

**Keywords:** Physics, Theoretical physics

## Abstract

In contemporary physics, the model of space–time as the fundamental arena of the universe is replaced by some authors with the superfluid quantum vacuum. In a vacuum, time is not a fourth dimension of space, it is merely the duration of the physical changes, i.e. motion in a vacuum. Mass–energy equivalence has its origin in the variable density of the vacuum. Inertial mass and gravitational mass are equal and both originate in the vacuum fluctuations from intergalactic space towards stellar objects.

## Introduction

The superfluid quantum vacuum model is replacing space–time as the fundamental arena of the universe^1–3^. In the superfluid vacuum (from now on ‘vacuum’) time is the numerical sequential order of material changes, i.e. motion running in a vacuum. The vacuum is timeless in the sense that time is not its fourth dimension^4^. The vacuum is the direct information medium of entanglement regarding EPR-type experiments: ‘Today, mainstream science considers that the observer and all observed physical phenomena exist in time and space. Nonetheless, recent research shows that the time measured with clocks is merely a mathematical parameter of material change, i.e. motion which runs in space. In this picture, the existence of past, present and future is merely a mathematical one. As regards EPR-type experiments, observer and observed phenomena exist only in space which originates from a fundamental quantum vacuum which is an immediate medium of quantum entanglement’^5^.

The formula for the variable density of the vacuum is defined by the mass and volume of a given stellar object. Let us imagine an ideal stellar object with mass *m* that is 93 billion light-years distant from other stellar objects, which is the diameter of today's observable universe. At the distance of 93 billion light-years from this ideal stellar object, we can assume that the density of the vacuum has a maximum value *ρ*_max_. On a stellar object's surface, the density of the vacuum is at the minimum (*ρ*_min_). The difference between these two densities is Δ*ρ*. A given ideal stellar object has diminishing density of vacuum on its surface exactly for the amount of its mass *m*. Considering that inertial mass *m*_*i*_ and gravitational mass *m*_*g*_ are proportional to the mass *m* as the amount of energy which is incorporated in a given stellar object, we can write the following equation:

1 $${m}_{i}={m}_{g}=m=({\rho }_{max}-{\rho }_{min})\cdot V,$$

where *V* is the volume of the physical object. The vacuum density difference Δ*ρ* is the source of permanent vacuum fluctuations in the direction from *ρ*_max_ towards *ρ*_min_. Inertial mass *m*_*i*_ and gravitational mass *m*_*g*_ of a given ideal stellar object both have their origin in these vacuum fluctuations (from now on **VF**), see Figs 1 and 2 below:

**Figure 1:** Vacuum fluctuations as the origin of inertial mass and of gravitational mass.

The article "Mass–Energy Equivalence Extension onto a Superfluid Quantum Vacuum" was retracted in 2021. Reasons: concerns about the data; concerns about the results or conclusions; concerns about the citations.

**Figure 2:** The density of the vacuum and vacuum fluctuations **VF**.

Density of the vacuum on the surface and of the stellar object we can calculate with the rearranging the Equation (1) as follows:

2 $${\rho }_{min}={\rho }_{max}-\frac{m}{V},$$

where *ρ*_min_ is the density of the vacuum on the surface of the stellar object.

Density of the vacuum at the distance *d* from the stellar object surface is following:

3 $${\rho }_{min}={\rho }_{max}-\frac{3m}{4\pi \cdot {(r+d)}^{3}},$$

where *r* is radius of the stellar object. When *d* is going towards the infinite, *ρ*_min_ becomes *ρ*_max_.

Inside the stellar object, the density of the vacuum *ρ* is increasing by the Newton shell theorem (see Fig. 2). At the distance *r* from the centre, the density of the vacuum, *ρ*, is the following:

4 $$\rho ={\rho }_{min}+\frac{3{m}_{1}}{4\pi \cdot {r}^{3}},$$

where *m*_1_ is the mass of the stellar object inside the shell and *r* is the radius of the shell. By increasing the vacuum density towards the centre of the stellar object, vacuum fluctuations are moving from the centre to the surface of the stellar object. Inside physical objects, we have two movements of vacuum fluctuations. One is from above towards the centre: *VF*_→_. The other is from the centre to the surface: *VF*_←_. These vacuum fluctuations are characteristic from the macro scale of the stellar objects to the micro scale of the proton.

## Vacuum Fluctuations, Binding and Repulsive Pressure of the Proton, Casimir Forces, and Van Der Waal Forces

Recent research confirms a strong repulsive pressure near the centre of the proton (up to 0.6 femtometres) and a binding pressure at greater distances^6^. In the model presented here vacuum fluctuations *VF*_→_ create binding pressure of the proton. Vacuum fluctuations *VF*_←_ create repulsive pressure of the proton (see Fig. 3 below).

**Figure 3:** Binding and repulsive pressure of the proton as the result of vacuum fluctuations **VF**.

Different authors are differently describing the Casimir effect: “The Casimir force^1^ is widely viewed as a force that originates from the vacuum energy, which is a view especially popular in the community of high-energy physicists^2–6^. Another view, more popular in the condensed-matter community, is that Casimir force has the same physical origin as van der Waals force^7–13^, which does not depend on energy of the vacuum. From a practical perspective, the two points of view appear as two complementary approaches, each with its advantages and disadvantages^7^”. In the model presented here, vacuum fluctuations *VF*_→_ are the origin of the Casimir effect when we have attraction force between plates. Repulsive forces between the plates are originated by vacuum fluctuations *VF*_←_. Also, van der Waals force can be described by vacuum fluctuations.

The article "Mass–Energy Equivalence Extension onto a Superfluid Quantum Vacuum" was retracted in 2021. Reasons: concerns about the data; concerns about the results or conclusions; concerns about the citations.

Recent research suggests there is no difference between Kasimir and van der Waal forces: “In fact, there are no two different forces, van der Waals and Casimir. The van der Waals force is a subdivision of dispersion forces acting at very short separations up to a few nanometers, where the effect of relativistic retardation is very small and can be neglected. As to the Casimir force, it is a subdivision of dispersion forces which acts at larger separation distances, where the effect of relativistic retardation should be taken into account. It is evident that there is some transition region between the two kinds of dispersion forces^8^”.

## Vacuum Fluctuations are the Origin of Gravity

Gravity force from the macro- to the microscale (proton) is the result of vacuum fluctuations **VF** as we can see in Fig. 4 below:

**Figure 4:** Gravity as the result of vacuum fluctuations **VF**.

The gravity force between physical objects is immediate. It does not require time and motion as is the case with photon propagation in space. The gravity force *F*_*g*_ between an object with mass *m*_1_ and an object with mass *m*_2_ is expressed by the following equation:

5 $${F}_{g}=\frac{{m}_{g1}\cdot {m}_{g2}\cdot G}{{r}^{2}},$$

where *m*_*g*1_ is the gravitational mass of the first object, *m*_*g*2_ is the gravitational mass of the second object. *m*_*g*1_ and *m*_*g*2_ are the result of vacuum fluctuations **VF** according to formula (1).

In General Theory of Relativity gravity is carried by the curvature of space. A given physical object is curving the space and curvature of space is generating gravity. In the model presented here vacuum is the physical origin of space. The variable density of space is generating vacuum fluctuations **VF** which are generating gravity. In both models, gravity is the result of properties of space (geometrical and physical properties) and is not acting directly between two physical objects.

NASA research confirms universal space is ‘flat’, it has a Euclidean shape, with only a 0.4% margin of error^9^. NASA results are suggesting that curvature of space in General Relativity is only the mathematical description of its actual density, which means the density of vacuum which is the physical origin of space. The curvature of space has only a mathematical existence and cannot carry gravity. The physical origins of gravity are vacuum fluctuations.

The article "Mass–Energy Equivalence Extension onto a Superfluid Quantum Vacuum" was retracted in 2021. Reasons: concerns about the data; concerns about the results or conclusions; concerns about the citations.

The idea of quantum gravity theory is that gravity is carried by some quanta: “Quantum gravity has been conjectured for almost 80 years since the introduction of the graviton. It is commonly believed that gravity is a fundamental interaction and as such, it would obey quantization similar to electrodynamics. However, it is significant to point out that there is not a single observational evidence so far showing the need of a quantum theory of gravity^10^”. In the model presented in this article gravity is not quantum phenomena. Gravity is the result of vacuum fluctuations *VF*_→_ which are generated by the presence of a given physical object.

## Vacuum Fluctuations and Gravitational Potential

The strength of vacuum fluctuations **VF** which generate inertia and gravity we express by gravitational potential. Gravitational potential *V* depends on the difference between the density of the vacuum in interstellar space and the density of the vacuum at the given point T, see Figs 5 and 6.

**Figure 5:** Gravitational potential and variable density of the vacuum.

**Figure 6:** Proton’s variable density of vacuum and Higgs potential.

At an infinite distance from a given stellar object, the gravitational potential *V* is zero, the density of the vacuum has its maximum value. At point T1, the gravitational potential *V* value is calculated by formula (6) below:

6 $$V=-\,\frac{GM}{r},$$

where *r* is the distance from the centre of the stellar object, *G* is the gravitational constant and *M* is the mass of the stellar object. On the stellar object surface at point T2, gravitational potential is calculated by formula (6). Inside the stellar object at point T3, we calculate the gravitational potential with the formula below:

7 $$V=-\,GM(\frac{3{R}^{2}-{r}^{2}}{2{R}^{3}}).$$

where *R* is the distance from the centre to the point T3^11^. In the centre of the stellar object at the point T4, *r* is zero, *R* is zero and the gravitational potential *V* is zero too.

## Mass–Energy Equivalence Extension onto the Vacuum

The gravity force at the points T1, T2, T3 (see Fig. 4) is always there in the form of vacuum fluctuations. If there is no physical object at the points T1, T2, T3 their gravity forces have no physical object to act upon, but they are there. Both inertia and gravity are the result of vacuum fluctuations, which have their origin in the variable density of the vacuum.

The article "Mass–Energy Equivalence Extension onto a Superfluid Quantum Vacuum" was retracted in 2021. Reasons: concerns about the data; concerns about the results or conclusions; concerns about the citations.

The curvature of space in General Relativity is a mathematical description of the variable density of the vacuum. The more space is curved, the less dense is the vacuum. Most of the universal space has a maximum value of vacuum density, *ρ*_max_. The vacuum density is decreasing in the areas with galaxies where universal space is flat too. The vacuum is the physical origin of the universal space, which means we can see a variable density of vacuum as an actual variable density of space. There is a fundamental dynamics between a given physical object with mass *m* and variable energy of space which we can describe with the following equation:

8 $$\frac{E}{{c}^{2}}=m=({\rho }_{max}-{\rho }_{min})\cdot V(8),$$

where *E* is the energy of the vacuum that is incorporated in a given physical object, *m* is the mass of the object, *ρ*_max_ is the density of space in the intergalactic area, *ρ*_min_ is the density of space on the surface of the physical object and *V* is the volume of a given physical object. This fundamental dynamics is the origin of mass–energy equivalence, inertia and gravity.

For relativistic particles, as for example a relativistic proton, the relativistic energy is the following:

9 $$E=\gamma \cdot {m}_{0}{c}^{2}=({\rho }_{max}-{\rho }_{minR})\cdot V\cdot {c}^{2},$$

where *E* is the proton relativistic energy, *γ* is the Lorentz factor, *m*_0_ is the proton rest mass and *ρ*_min R_ is the density of the vacuum at the relativistic proton surface. The proton, when accelerated, is interacting with the vacuum and additionally incorporating some of its energy.

Fedi has developed a model of the vacuum as a shear-thickening (dilatant) fluid (the Newtonian fluid)^12^. In his model relativistic energy of the proton can be seen as accelerated proton thickens the vacuum ahead of it.

If the accelerated proton is absorbing the vacuum energy or is thickening the vacuum energy ahead of it remains an open question for now. Important is that both models see the relativistic energy of the proton as the energy of the vacuum which is absorbed or is thickening ahead of the proton. Proton does not gain its relativistic energy because of the motion in an empty space. Proton relativistic energy is vacuum energy which is interacting with the proton due to its motion in a vacuum.

## The Density of the Vacuum on the Black Hole Surface, Neutron Star Surface and Proton Surface

The density of the vacuum *ρ*_min_ on the surface of a black hole with the mass of the Sun and radius of 3000 metres is according to formula (4) the following:

$$\begin{array}{rcl}{\rho }_{{\rm{\min }}} & = & {\rho }_{{\rm{\max }}}-\frac{1.989\cdot {10}^{30}\,kg}{1,131\cdot {10}^{11}\,{m}^{3}}\\ {\rho }_{{\rm{\min }}} & = & {\rho }_{{\rm{\max }}}-1.759\cdot {10}^{19}\,kg/{m}^{3}\end{array}$$

The density of the vacuum *ρ*_min_ on the surface of planet Earth is given by the following:

$$\begin{array}{rcl}{\rho }_{{\rm{\min }}} & = & {\rho }_{{\rm{\max }}}-\frac{5.972\cdot {10}^{24}\,kg}{1,083\cdot {10}^{21}\,{m}^{3}}\\ {\rho }_{{\rm{\min }}} & = & {\rho }_{{\rm{\max }}}-5.514\cdot {10}^{3}\,kg/{m}^{3}\end{array}$$

The density of the vacuum *ρ*_min_ on the surface of the proton is given by the following:

$$\begin{array}{rcl}{\rho }_{{\rm{\min }}} & = & {\rho }_{{\rm{\max }}}-\frac{1.672\cdot {10}^{-27}\,kg}{2.5\cdot {10}^{-45}\,{m}^{3}}\\ {\rho }_{{\rm{\min }}} & = & {\rho }_{{\rm{\max }}}-6.688\cdot {10}^{17}\,kg/{m}^{3}\end{array}$$

The density of the vacuum on the surface of a neutron star is ${\rho }_{{\rm{\min }}}={\rho }_{{\rm{\max }}}-2.0\cdot {10}^{26}\,kg/k{m}^{3}$ ^13^, which is ${\rho }_{{\rm{\min }}}={\rho }_{{\rm{\max }}}-2.0\cdot {10}^{17}\,kg/{m}^{3}$.

The article "Mass–Energy Equivalence Extension onto a Superfluid Quantum Vacuum" was retracted in 2021. Reasons: concerns about the data; concerns about the results or conclusions; concerns about the citations.

Regarding the maximum density *ρ*_max_ which is constant, the density of the vacuum *ρ*_min_ on the surface of the black hole is of the order −10^19^. Regarding the maximum density *ρ*_max_, the density of the vacuum *ρ*_min_ on the surface of the proton is of the order −10^17^. Regarding the maximum density *ρ*_max_, the density of the vacuum *ρ*_min_ on the surface of the neutron star is of the order −10^17^. Regarding the maximum density *ρ*_max_, the density of the vacuum *ρ*_min_ on the surface of the planet Earth is of the order −10^3^.

Recent research results are that the average peak pressure near the centre of the proton is about 10^35^ pascals, which exceeds the pressure estimated for the most densely packed known objects in the universe, neutron stars^6^. The calculations above confirm minimal density of the vacuum on the proton surface is ${\rho }_{{\rm{\min }}}={\rho }_{{\rm{\max }}}-6.688\cdot {10}^{17}\,kg/{m}^{3}$. Minimal density of the vacuum on the neutron star surface is ${\rho }_{{\rm{\min }}}={\rho }_{{\rm{\max }}}-2.0\cdot {10}^{17}\,kg/{m}^{3}$. Density of the vacuum on the proton surface is smaller from the density of the vacuum on a neutron star surface. That is why the peak pressure near the centre of the proton exceeds the peak pressure in neutron stars.

The density of the vacuum on the surface of a proton is ${\rho }_{{\rm{\min }}}={\rho }_{{\rm{\max }}}-6.688\cdot {10}^{17}\,kg/{m}^{3}$. The density of the vacuum on the surface of a black hole is ${\rho }_{{\rm{\min }}}={\rho }_{{\rm{\max }}}-1.759\cdot {10}^{19}\,kg/{m}^{3}$. On the surface of a black hole, the density of the vacuum is too low to keep a proton stable. Protons are falling apart and disintegrating back into the energy of the vacuum. This reduces the mass and the energy of the black holes^14^.

The article "Mass–Energy Equivalence Extension onto a Superfluid Quantum Vacuum" was retracted in 2021. Reasons: concerns about the data; concerns about the results or conclusions; concerns about the citations.

Steven Hawking predicted that the mass and energy of a black hole are diminishing because of thermal radiation, also known as black hole evaporation^15^. A recent article has reported the observation of quantum Hawking radiation in an analogue black hole^16^. Another recent article raises severe doubts about the observation of Hawking radiation^17^.

The proton rest mass is *m*_0_ = 1.672 ⋅ 10^−27^ *kg*. In an accelerator, the proton relativistic energy reaches in terms of rest mass *m*_0_ a value of *E* = *m*_0_ ⋅ *c*^2^ ⋅ 7460. When this relativistic energy would be considered as mass, the relativistic proton would become a mini black hole. The relativistic energy of the accelerated proton is the energy of the vacuum, which is additionally integrated into the proton. Comparing with the mass of the black hole, we cannot consider the relativistic energy of the proton as a mass. Mass of the black hole is the mass of the stellar object which is moving in the universal space far beyond the velocity of the light speed and relativistic energy of the proton is the result of its ecceleration close to the light speed. This means that the existence of mini black holes predicted by Stephen Hawking^18^ is questionable. Voyager data excludes the existence of mini black holes^19^.

## Variable Vacuum Density and Variable Rate of Clocks

What is the value of vacuum density *ρ*_max_ (which when multiplied by *c*^2^ becomes vacuum energy density) is a big dispute in today’s physics: ‘The theoretical vacuum energy density estimated on the basis of the Standard Model of particle physics and very general quantum assumptions is 59 to 123 orders of magnitude larger than the measured vacuum energy density for the observable universe which is determined on the basis of the Standard Model of cosmology and empirical data. This enormous disparity between the expectations of two of our most widely accepted theoretical frameworks demands a credible and self-consistent explanation, and yet even after decades of sporadic effort, a generally accepted resolution of this crisis has not surfaced’^20^.

In this article the subject of vacuum density remains open. Some theoretical research speculates the vacuum might be a four-dimensional reality: ‘It is a general trend in modern theoretical physics to consider extended objects, like strings and membranes. Usually, one applies these ideas to hypothetical, high-dimensional completions of the four-dimensional world. However, lower-dimensional structures might also exist in four dimensions. At the present time, there is no well-developed theory which would predict such structures. However, there is accumulating evidence obtained within the lattice QCD that there are lower dimensions objects percolating through the vacuum of four-dimensional Yang–Mills theories’^21^. Some other researchers predict the vacuum could be a four-dimensional reality^22,23^. If the vacuum actually is four dimensional, we cannot apply a classical understanding of vacuum density, which works only in the three-dimensional domain.

The article "Mass–Energy Equivalence Extension onto a Superfluid Quantum Vacuum" was retracted in 2021. Reasons: concerns about the data; concerns about the results or conclusions; concerns about the citations.

Rather, I will show the relatedness between the variable density of the vacuum and the variable rate of clocks. With a variable rate of clocks, we can indirectly measure the variable density of the vacuum. In General Relativity, the gravitational time dilation is calculated using the following formula:

10 $$t=\frac{{t}_{0}}{\sqrt{1-\frac{2GM}{r{c}^{2}}}},$$

where *t*_0_ is the rate of the clock on the surface of the stellar object, *M* is the mass of the stellar object, *G* is the gravitational constant, *r* is the radius of the stellar object and *t* is the rate of the clock at the point *T* which is infinitely away in empty cosmic space. For example, when one second has passed on the Earth surface, at the point *T* in infinity 1.000000000695915 second has passed. We can calculate the rate of a clock at point *T*_1_, situated at the distance *h* above the surface of the stellar object with the following formula:

11 $$t={t}_{0}\cdot \sqrt{\frac{1-\frac{2GM}{(r+h)\cdot {c}^{2}}}{1-\frac{2GM}{r{c}^{2}}}}.$$

Let us calculate the time *t* at a point 20 km above the Earth’s surface comparing with the 1 second elapsed time on the Earth’s surface:

$$\begin{array}{rcl}t & = & 1s\cdot \sqrt{\frac{1-\frac{2(5.97219\times {10}^{24}\,kg)(6.67408\times {10}^{-11}\,{m}^{3}k{g}^{-1}{s}^{-2})}{(6371000m+20000m)(8.99\times {10}^{16}\,{m}^{2}{s}^{-2})}}{1-\frac{2(5.97219\times {10}^{24}\,kg)(6.67408\times {10}^{-11}\,{m}^{3}k{g}^{-1}{s}^{-2})}{(6371000\,m)(8.99\times {10}^{16}\,{m}^{2}{s}^{-2})}}}\\ t & = & 1s\cdot \sqrt{\frac{1-0.00000000138747}{1-0.00000000139183}}\end{array}$$

$$t=1.00000000000218s\,(20\,\text{km above the surface}).$$

Let us calculate the time *t* at the point 40 km above the Earth’s surface compared with the 1 second elapsed time on the Earth’s surface:

$$\begin{array}{rcl}t & = & 1s\cdot \sqrt{\frac{1-\frac{7.9717748\times {10}^{14}\,{m}^{3}{s}^{-2}}{(6411000m)(8.99\times {10}^{16}\,{m}^{2}{s}^{-2})}}{1-\frac{7.9717748\times {10}^{14}\,{m}^{3}{s}^{-2}}{(6371000m)(8.99\times {10}^{16}\,{m}^{2}{s}^{-2})}}}\\ t & = & 1s\cdot \sqrt{\frac{1-0.00000000138315}{1-0.00000000139183}}\end{array}$$

$$t=1.00000000000434s\,(40\,\text{km above the surface}).$$

Let us calculate the time *t* at the black hole with the mass of the Sun and radius of 3000 metres compared with the elapsed *t*_∞_ = 1,000000000695915*s*:

$$\begin{array}{rcl}{t}_{\infty } & = & \frac{{t}_{black\mbox{--}hole}}{\sqrt{1-\frac{2GM}{r{c}^{2}}}}\\ {t}_{black\mbox{--}hole} & = & 1.000000000695915s\cdot \sqrt{1-\frac{2\cdot 1,989\cdot {10}^{30}kg\cdot 6.67408\cdot {10}^{-11}\,{m}^{2}k{g}^{-1}{s}^{-2}}{3\cdot {10}^{3}\cdot 8.99\cdot {10}^{16}\,{m}^{2}{s}^{-2}}}\\ {t}_{black\mbox{--}hole} & = & 1.000000000695915s\cdot \sqrt{1-0.98440824026696}\\ {t}_{black\mbox{--}hole} & = & 0.12486696822s\end{array}$$

Black hole surface *t*_*black*–*hole*_ = 0.12486696822*s*.

The article "Mass–Energy Equivalence Extension onto a Superfluid Quantum Vacuum" was retracted in 2021. Reasons: concerns about the data; concerns about the results or conclusions; concerns about the citations.

Earth surface *t*_0_ = 1*s*.

20 km above Earth surface *t*_20_ = 1.00000000000218*s*.

40 km above Earth surface *t*_40_ = 1.00000000000434*s*.

Infinite distance from Earth surface *t*_∞_ = 1.000000000695915*s*.

The rate of clocks is increasing with increasing vacuum density. Where the density of the vacuum is at the maximum *ρ*_max_, the rate of clocks is at the maximum too. With the diminishing of vacuum density, the rate of clocks is diminishing. The General Relativity effect causes clocks on the GPS satellites to run faster than on the Earth’s surface by 45 microseconds per day^24^. This is because on the satellite trajectory the vacuum is denser than on the Earth’s surface.

GPS satellites are moving with a velocity *v* with respect to the Earth’s surface. Because of its kinetic energy, the mass *m* of a given satellite is increasing:

12 $$m={m}_{0}+\frac{{m}_{0}{v}^{2}}{2{c}^{2}},$$

where *m*_0_ is the mass of the satellite on the Earth’s surface, *v* is the velocity of the satellite relative to the Earth’s surface. Because of the increased mass *m* of the moving satellite, the density of vacuum inside the satellite additionally decreases. The decrease of vacuum density causes clocks to run slower on the satellite than on the Earth’s surface. The value of this Special Relativity effect is 7 microseconds per day^24^.

The variable rate of clocks is directly related to the variable vacuum density. We could numerically evaluate the vacuum density on the surface of a given stellar object by considering that the numerical value of the vacuum infinitely distant from the stellar object is *ρ*_∞_ = 1.000000000695915. On the Earth’s surface the numerical value of vacuum density is *ρ*_*earth*_ = 1. On the black hole surface the numerical value of vacuum density *ρ*_*black*–*hole*_ = 0.12486696822.

In 20^th^ century physics, the unsolved question was whether inertial mass and gravitational mass are caused by the mass of the given stellar object or are related to the masses of other stellar objects in the universe: ‘If the rest of the universe determines the inertial frames, it follows that inertia is not an intrinsic property of matter, but arises as the result of matter with the rest matter of the universe. This immediately raises the problem of how Newton's laws of motion can be accurate despite their complete lack of reference to the physical properties of the universe, such as the amount of matter it contains’^25^. The results of this research confirm that inertial mass and gravitational mass of a given stellar object with the mass *m* have their origin only in its mass, which causes the variable density of vacuum Δ*ρ*, see Equation (2), and are not related to the masses of other stellar objects.

The article "Mass–Energy Equivalence Extension onto a Superfluid Quantum Vacuum" was retracted in 2021. Reasons: concerns about the data; concerns about the results or conclusions; concerns about the citations.

## The Variable Density of Vacuum in Proton and Higgs potential

In this chapter variable density of vacuum will be interpreted as the Higgs potential. Recent research presents the Higgs potential as follows: “The Higgs potential *V*(*H*) for a simple case of a real scalar field *H* can be written as:

13 $$V(H)=\lambda {({H}^{2}-{v}^{2})}^{2}=\lambda {H}^{4}-2\lambda {v}^{2}{H}^{2}+\lambda {v}^{4},$$

where *H* is the Higgs field^26^. Both *v* and *λ* paramaters are determined experimentally through the measurement of the Fermi constant *GF* and the Higgs boson mass *MH* = 125 *GeV*, yielding *v* = 246 *GeV*, *λ* = 0,13. *V*(*H*) can be interpreted as the Higgs vacuum energy density (energy density of the empty space). For our choice of the potential, the vacuum energy density is zero at the minimum *H* = *v*. However, for the potential energy it is the difference that matters, not the absolute value and thus the relevant contribution is the constant term in Eq. 24 (the size of the hill at *H* = 0), *λv*^4^ = 4.8⋅10^8^ *GeV*^4^. From cosmology we have a vacuum energy density that is roughly 55 orders smaller and this huge difference is a mystery, the cosmological constant problem^26^.

In the model here presented density of the vacuum in interstellar space has the value of *ρ*_max_. We do not know yet the actual value of *ρ*_max_ which presents the actual cosmological constant problem. 5% of the energy in the universe is ordinary matter. The 65% percent is missing dark energy and 27% is missing dark matter. Considering that universal space has its physical origin in the vacuum, the energy of the vacuum itself can be the missing dark energy and the missing dark matter. The energy of the vacuum is not interacting with the light and remains invisible and undetectable.

The idea of 20^th^-century physics was that stellar objects exist in an empty space deprived of physical properties. This idea has led to the prediction of dark energy and dark matter. With the introduction of the vacuum which has variable density the question of dark energy and dark matter is seen from the new perspective which is promising to advance the solution for the cosmological constant problem. On the other hand, considering that vacuum could be a four-dimensional reality^21–23^, the density of the vacuum could remain an open subject for a longer period of time because density (or energy density) is seen in today physics as three-dimensional phenomenon.

The article "Mass–Energy Equivalence Extension onto a Superfluid Quantum Vacuum" was retracted in 2021. Reasons: concerns about the data; concerns about the results or conclusions; concerns about the citations.

The idea that vacuum energy density is zero at the minimum *H* = *v*^26^ is questionable. If we define vacuum energy density value is zero, then universal space could not exist anymore, because the vacuum is the physical origin of the universal space. The vacuum is the physical origin of the universal space; vacuum energy density (or density in the model presented in this article) is variable and bigger than zero in entire universal space.

The model presented in this article suggests that minimal vacuum density *ρ*_min_ on the surface of the proton placed in interstellar space is at the bottom of the hat, the density of vacuum in the centre of the proton *ρ*_*centre*_ is on the top of the hat, the density of the vacuum away from the proton *ρ*_max_ is on the edge of the hat (see Fig. 6).

In the proton, vacuum fluctuations are moving from the *ρ*_max_ to the *ρ*_min_, and from the *ρ*_*centre*_ to the *ρ*_min_. These vacuum fluctuations are the physical origin of the Higgs potential.

The superfluid quantum vacuum model with the variable density is the development of the electromagnetic quantum vacuum model (QED) which is one of the most successful theories. With giving electromagnetic vacuum variable density as presented in this article, we can describe Higgs potential and also the origin of gravity. The perspective of further research on the variable density of vacuum is to integrate QED with the Higgs mechanism model and quantum gravity model.

Recent research of Sbitnev on the hydrodynamics of the physical vacuum^1^ opens the new perspective where elementary subatomic particles could be seen as the vacuum vortexes. In Sbitnev model the vortex is periodically exchanging energy with the vacuum via vacuum fluctuations. Sbitnev model is enhancing the model of vacuum fluctuations presented in this article with clear insight, namely, we cannot study subatomic particles without considering their active relatedness with the vacuum.

According to the model presented in this article, a given vortex is in active relation with the vacuum. When accelerated the vortex is “dragging” with the vacuum and absorbing some of its energy which is its relativistic energy.

The article "Mass–Energy Equivalence Extension onto a Superfluid Quantum Vacuum" was retracted in 2021. Reasons: concerns about the data; concerns about the results or conclusions; concerns about the citations.

Considering that vacuum is 4-dimensional^21–23^, and so proton is 4-dimensional vacuum vortex, we are limited in the proton observation with the 3-dimensional apparatuses and 3-dimensional sensorial sense (sight). Taking into account that atom is three dimensional, the subatomic world could be four and more dimensional. We have to be aware that higher dimensionality of the subatomic world represents the limitation of our scientific endeavor.

## Conclusions

When modelling mass–energy equivalence, inertia and gravity, we cannot develop an objective model without considering that space has physical properties. With the introduction of the superfluid quantum vacuum, which is the physical origin of the universal space, the new perspective presented in this article is open. This model confirms that inertial mass and gravitational mass are equal and both have their origin in the vacuum fluctuations caused by the variable density of vacuum.
